# Biomarkers for Breast Adenocarcinoma Using In Silico Approaches

**DOI:** 10.1155/2022/7825272

**Published:** 2022-03-03

**Authors:** Jhansi Pandi, Ajucarmelprecilla Arulprakasam, Ranjithkumar Dhandapani, Saikishore Ramanathan, Sathiamoorthi Thangavelu, Jayaprakash Chinnappan, V. Vidhya Rajalakshmi, Saad Alghamdi, Nashwa Talaat Shesha, S. Prasath

**Affiliations:** ^1^Medical Microbiology Unit, Department of Microbiology, Alagappa University, Karaikudi, Tamil Nadu, India; ^2^Chimertech Private Limited, Chennai, India; ^3^Department of Bioinformatics, Bharathiar University, Coimbatore, Tamil Nadu, India; ^4^Laboratory Medicine Department, Faculty of Applied Medical Sciences, Umm Al-Qura University, Makkah, Saudi Arabia; ^5^Hera General Hospital, Directorate of Health Affairs, Makkah, Saudi Arabia; ^6^Department of Mechanical Engineering, College of Engineering and Technology, Mizan Tepi University, Ethiopia

## Abstract

This work elucidates the idea of finding probable critical genes linked to breast adenocarcinoma. In this study, the GEO database gene expression profile data set (GSE70951) was retrieved to look for genes that were expressed variably across breast adenocarcinoma samples and healthy tissue samples. The genes were confirmed to be part of the PPI network for breast cancer pathogenesis and prognosis. In Cytoscape, the CytoHubba module was used to discover the hub genes. For correlation analysis, the predictive biomarker of these hub genes, as well as GEPIA, was used. A total of 155 (85 upregulated genes and 70 downregulated genes) were identified. By integrating the PPI and CytoHubba data, the major key/hub genes were selected from the results. The KM plotter is employed to find the prognosis of those major pivot genes, and the outcome shows worse prognosis in breast adenocarcinoma patients. Further experimental validation will show the predicted expression levels of those hub genes. The overall result of our study gives the consequences for the identification of a critical gene to ease the molecular targeting therapy for breast adenocarcinoma. It could be used as a prognostic biomarker and could lead to therapy options for breast adenocarcinoma.

## 1. Introduction

Breast malignancy or bosom cancer is the most widely recognized sort of malignancy, particularly among women. Main causes for breast cancer were hereditary predisposition, changes in hormonal levels, multifactorial, and implicated reproductive factors [1]. Currently, the majority of women experience breast malignancy, also known as bosom (breast area of the body) malignant growth, and the fatality rate is common among women. Bosom malignant growth is majorly caused by lifestyle changes like diet and cell phone exposure directly to the breast area, and due to hereditary changes [2, 3]. BRCA1 and BRCA2 were found to be significant genes related to hereditary breast malignancy. BRCA1 and BRCA2 were situated on chromosome 17 and chromosome 13, respectively, where a mutation in either of these two genes deliberates the increased risk of breast cancer [4]. Before the time, cervical disease was the most widely recognized malignancy in India, and currently breast cancer is more noteworthy than cervical malignancy and turned into a main malignancy that causes ductal carcinoma in situ, obtrusive ductal carcinoma, and fiery bosom disease [5]. By 2020, BC became the most well-known malignancy analyzed among ladies rather than men, surpassing lung cancer, estimating 2.3 million newly diagnosed cases. Under 0.2% of malignant growth-related mortality in women can be credited to breast cancer. Death rates of breast cancer were considerably high followed by cervical cancer [6, 7]. Some of the hazardous risk factors of breast malignancy incorporate age, early menarche, childbearing, late menopause, diet, burning-through of liquor, smoking, family history, low breastfeeding for a limited period, history of premature delivery, purposeful weight reduction, chest X-beam, BMI, type 2 diabetes, bosom thickness, utilization of oral prophylactic, and chemical substitution therapy [8, 9].

Due to high cost and financial, geological, and social obstacles associated to women's health, there is a lack of knowledge regarding breast cancer indicators and diagnosis is a key factor for the late conclusion of sickness poor treatment [10]. Detection of breast cancer by digital bosom tomosynthesis (DBT) is an ordinary mammographic procedure, which, as of the late improved strategy, gives a semi-3-dimensional picture of the bosom. Bosom attractive reverberation imaging (MRI), abbreviated bosom MRI (AB-MR), and whole-bosom ultrasound are utilized for the analysis of breast adenocarcinoma [11]. Treatment for breast adenocarcinoma includes a mixture of medical procedures, radiotherapy, and hormonal treatment. The tumor-related factors like size, grade, and mitotic rate and medical procedure, extent of surgery, width of edge radiation, and utilization of tamoxifen could affect the ipsilateral rate of events after DCIS treatment. The principle of this treatment is the disposal of the sickness [12]. The treatment options incorporate medical procedure, radiotherapy, chemotherapy, or chemical treatment. It relies upon the expectation, phase of infection, antagonistic impacts, and therapy options [13]. DCIS (ductal carcinoma in situ) and invasive breast carcinoma both have many similarities regarding morphology and molecular level. However, in differentiating the above two different lesions, MEC layer and the surrounding BM come into display [14]. The maximum normally used molecular-centered drugs for HER2-positive breast cancer consist of tucatinib, trastuzumab, pertuzumab, lapatinib, neratinib, and trastuzumab emtansine (T-DM1). Several pills target the phosphoinositide-3-kinase (PI3K)/serine/threonine kinase (AKT)/mammalian target of rapamycin (mTOR) signaling pathways, including GDC-0068, Bez235, bupacoxib, abencoxib, and alpelisib. Vascular endothelial growth factor (VEGF) has also been identified as a key target for antiangiogenic remedy, and its inhibitors sorafenib, sunitinib, and bevacizumab are also used for breast cancer therapy. However, due to tumor heterogeneity, low ratios of responders, and relapse, there is an urgent need to perceive new biomarkers, which can usefully resource the analysis and treatment of breast cancer [15].

This study illuminates the idea of identifying the probable therapeutic biomarkers that were linked to breast adenocarcinoma. In this work, a gene expression profile with accession number GSE70951 is selected from the GEO database in which Gene Expression Omnibus informational index provides much information about microarray experiment data sets. GEO2R was used to determine DEGs, and bioinformatics analysis such as biological processes, molecular functions, and cellular components in gene ontology and enrichment pathway analysis were carried out. A PPI network was built for recognizing the center quality of the outcome. For finding the correlation of hub genes and expression level, the KM plotter was used for survival analysis and GEPIA was used for correlation analysis. Finally, several breast cancer-related molecules have been selected to investigate their potential role in a breast cancer diagnostic system. The above study might contribute in understanding the mechanism of potential biomarkers identified for breast adenocarcinoma.

## 2. Materials and Methods

### 2.1. Data Sources

The GEO database is a public repository, which contains microarray data and next-generation sequencing data for further analysis. One gene expression profile (GSE70951) from the GEO data collection was used in this study since it was concentrated in previous studies, contributed by Quigley et al., with GPL4133 and GPL13607 being the platforms. GPL4133 stage, for example, relied on Agilent-014850 Whole Human Genome Microarray 4 × 44k G4112 F. Agilent-028004 SurePrint G3 Human GE 8 × 60k Microarray was required for GPL13607. GSE70951 containing 433 samples were chosen for a consecutive study along with the following criteria: DEGs between breast adenocarcinoma and normal surrounding tissue were investigated using the *R* language in limma package.

### 2.2. Analysis of DEGs through Enrichr

Gene ontology and enrichment pathway analyses were performed to clarify the potential functions of the variably expressed genes. Enrichr, a recently released online tool for enrichment analysis, is an important component of high-throughput gene function investigation. BP, CC, and MF are the three categories of gene function prediction. KEGG is widely used to contain enormous data information about biological pathways, genomes, diseases, chemical compounds, and medications and integrated with modules and networks.

### 2.3. PPI and Module Analysis

STRING is used to construct a PPI network for DEGs with a high confidence score of 0.700 as the cutoff criterion, and repeated linkages were deleted in the current study. The networks were directed with plug-in CytoHubba, which is a component tool in Cytoscape software, version 3.8.2. Hub genes were identified based on the highest degree score from the protein-protein interaction result. The plug-in MCODE application was used to find the clustering nodules of hub genes in the PPI network. Hub genes were defined with at least 10 gene degrees in the PPI network, and all those network diagrams of key genes were visualized with Cytoscape software (version 3.8.2).

### 2.4. Survival Analysis of Hub Genes

The survival analysis was performed to examine the prognostic impact of 10 genes in BAC patients through the KM plotter. In breast cancer, the Kaplan–Meier plotter was used to investigate the prognostic benefits of every single pivot gene. According to these overall survival details, the genes were sorted from high to low expression based on the TCGA database. The *P* value log rank was determined and shown in the site page, as well as with 95% of the confidence intervals in HR (hazard ratio).

### 2.5. Analysis of Correlation and Expression Levels

GEPIA is used to detect the levels of expression and correlation analysis of the hub genes. It provides a normal vs. tumor differential expression as a box plot. The box plot shows the visualization difference between the BAC tissue and normal tissue. TCGA-BRCA is used to confirm the expression of genes. Furthermore, the correlation analysis investigates the relative ratios between two genes using pairwise gene correlation analysis of TCGA expression data.  Figure 1 shows the overall work plan for identification of strong prognostic biomarker genes in BAC.

## 3. Results

### 3.1. Identification of DEGs

In this study, one of the most recent gene expression profiles (GSE70951) was taken. GPL4133 had 46 normal samples and 46 breast adenocarcinoma (BAC) samples, whereas GPL13607 had 147 normal samples and 147 BAC samples. By comparing BAC samples with normal samples (Table 1), all DEGs were discovered.

The DEGs are of the two sets of data that appear in the gene expression profiles displayed in the volcano plot (Figure 2) and heat map (Figure 3) Furthermore, Venn diagram analysis was used to determine the overlap in the middle of DEG profiles (Figure 4).

Finally, 155 DEGs were found to be differentially expressed between the two data sets, among them 85 being effectively upregulated and 70 being effectively downregulated genes (Table 2). By using the criteria |log^2^ FC| ≥ 1.0 and adjusted *p* value < 0.5, DEGs were acquired.

### 3.2. Analysis of Functional Enrichment in DEGs

In DEGs, Enrichr was used to analyze the pathway of KEGG enrichment and the function of gene ontology. The enriched GO elements were grouped based on BP, CC, and MF. The outcome analysis of gene ontology shows that DEGs are primarily enriched in the following processes:

1. In BP, L-phenylalanine metabolic process, aromatic amino acid family catabolic process, L-phenylalanine catabolic process, regulation of glial cell differentiation, and erythrose 4-phosphate/phosphoenolpyruvate family amino acid catabolic process were included.
2. In MF, the DEGs were highly enriched in choline transmembrane transporter activity, peptidyl-proline 4-dioxygenase activity, MHC class II protein binding, carbonate dehydratase activity, and organic cation transmembrane transporter activity.
3. In cellular components, the DEGs were abundant in meiotic cohesion complexes, condensed nuclear chromosomes, L-type voltage-gated calcium channel complex, condensed nuclear chromosome, kinetochore, centromeric region, and condensed nuclear chromosome G-protein coupled receptor dimeric complex.

The above analyses revealed that transcriptional activity, cell cycle regulation, binding, and cell proliferation are significantly enhanced in the majority of DEGs. These studies revealed that the DEGs were largely enriched in phenylalanine, tyrosine and tryptophan biosynthesis, ECM receptor interaction, nitrogen metabolism, phenylalanine metabolism, and IL–17 signaling pathway.

### 3.3. Selection of Hub Genes

The STRING database was utilized to recognize the differential gene expression between the PPI networks. In the PPI network (Figure 5), a total of 9 nodes and 20 edges were displayed below. The high connectedness degree in the top 10 genes was detected by PPI networks (Figure 6). The result shows that the mitotic checkpoint serine/threonine protein kinase BUB1 was the highly enriched gene, with the connectedness degree = 14, followed by non-SMC condensin I complex, subunit *G* (NCAPG, connectedness degree = 14), syndecan 1 (SDC1, connectedness degree = 14), Rac GTPase-activating protein 1 (RACGAP1, connectedness degree = 13), fibronectin 1 (FN 1, connectedness degree = 13), serine/threonine protein kinase chk1 (CHEK1, connectedness degree = 12), DEP domain-containing protein 1 A (DEPDC1, connectedness degree = 12), thymidylate synthase (TYMS, connectedness degree = 12), SHC SH2 domain-binding protein 1 (SCHB P1, degree = 11), and cell division cycle 7-related protein kinase (CDC7, connectedness degree = 10). All these hub genes were enhanced in breast adenocarcinoma.

### 3.4. Overall Survival for Key Genes

The KM plotter is used to analyze the survival of these 10 genes. The relationship between the expression levels of 10 genes and the risk of breast cancer metastasis was indicated by confidence interval and *p* value. (Table 3). In this study, these 10 hub genes show a worse survival rate in overall and confirm the prognostic value of BAC (Figure 7).

### 3.5. Validation of Key Genes

The above results were validated by detecting the expression levels of these top 10 pivot genes in the middle of BAC tumor samples and normal samples (Figure 8), and from that, when compared with normal tissue, the 10 hub genes are highly expressed and it is evident. The green color represents “tumor,” and the gray color represents “normal”. Those genes show higher expression levels than normal tissue. In correlation, the BUB1 gene had the most extensive level worth in the PPI network, for that reason BUB1 was selected for conducting the correlation analysis (Figure 9). Analysis of data from GEPIA in BUB1 had strongly correlated with other 7 (NCAPG, CHEK, RACGAP1, SHCBP1, CDC7, DEPDC1, and TYMS) hub genes, and among them NCAPG, RACGAP1, and DEPDC1 were strongly correlated with the coefficients 0.76, 0.71, and 0.7, respectively (Pearson *r* > 0.5 and *p* < 0.1), and these expressed genes do not assume a significant part in the forecast of BAC patients yet be essential in the movement and pathology of this illness. SDC1 and FN1 do not have a significant *p* value and scattered plots, and hence there is no correlation with BUB1. This shows the BUB1 hub gene's importance and interactivity with other BAC disease-related genes.

## 4. Discussion

Despite latest advancements in the treatment of breast cancer, it has been remained as the most common cause of cancer-related death in recent decades. The excessive mortality rate of bosom cancer is due to the dearth of adequate screening strategies with high sensitivity and specificity. Therefore, it is very necessary to discover highly capable biomarkers for screening and early diagnosis of bosom cancer. Microarray technology and subsequent-generation sequencing has become key tools for imparting comprehensive genetic statistics on bosom cancer samples and revealing the adjustments in sickness progression. In this study, the GEO database is used to download the microarray data (GSE70951—Paired Breast Adenocarcinoma and Adjacent Normal Tissue). 155 differentially expressed genes were reserved into categories by functional annotation, as well as gene ontology groups. The outcome of functional enrichment analysis shows that notably differentially expressed genes were involved in the L-phenylalanine metabolic process, regulation of glial cell differentiation, L-phenylalanine catabolic process, phosphoenolpyruvate family amino acid catabolic process, and aromatic amino acid family catabolic process. From the GEPIA database, it is found that BUB1, NCAPG, CHEK1, RACGAP1, SHCBP1, SDC1, CDC7, DEPDC1, TYMS, and FN1 were highly enriched in the PPI network with high degree values in BRCA samples. Survival analysis of these genes shows worse prognosis when performed in the KM plotter, and coincidentally these genes were overexpressed when compared with normal tissue. In addition, they do not have a pivotal role in the prognosis of BAC, but they do involve in the progression and pathology of this disease.

BUB1 kinase, a crucial spindle key checkpoint regulator, now has extra pleiotropic functions. By targeting the metaphase congression and Shugoshin protein, BUB1 is essential for the connection of a functioning inner centromere and sister chromatid cohesion. The presence of BUB1 mutation in colorectal tumors suggests that it could be a stimulant for carcinogenesis by causing chromosomal instability and aneuploidy [16]. NCAPG, cell cycle related, is a component of the condensing complex, according to prior studies; NCAPG is overexpressed in various types of tumors. Recent studies revealed that NCAPG knockdowns [R] have induced apoptosis, reduced the survival of cancer cells, and suppressed the EMT in cancer [17]. CHEK1 (checkpoint kinase 1) encodes a serine/threonine protein kinase, which synchronizes DNA damage response, a cell death pathway stimulator and involved in checkpoint activation [18]. Rac GTPase-activating protein 1 (RacGAP1) may result in several types of tumors including bosom cancer, gastric carcinoma, etc, due to the overexpression of RacGAP1. Transition in RacGAP1 may be associated with few malignancies such as hepatocellular carcinoma, meningioma, and epithelial ovarian cancer. Additionally, cell change and metastasis are associated with RacGAP1 [19]. SHCBP1 communicates with the connector protein Shc A and plays a significant part in cell division, cell growth, cell proliferation, and differentiation. SHCBP1 is essential for the completion of cytokinesis and organization of the midbody [20]. The gene SDC1 encodes syndecan 1 protein, which is a transmembrane heparan sulfate proteoglycan. This protein takes up a key role in the regulation including cell proliferation, adhesion, migration, and modulation of cell-matrix and cell-cell interactions during wound healing. Overexpression of SDC1 was found to be more frequent in bosom carcinoma than in NT and therefore might be considered as a potential biomarker of breast cancer. Additionally, the overexpression of the gene is considerably correlated with the increased risk of age, higher SBR grade status, nodal, and HER2 [21]. CDC7 (cell division cycle 7-related protein kinase) was involved in the cell cycle during DNA replication in the chromosome for maintaining replication forks [22]. DEPDC1 (DEP domain-containing 1 protein), which is a highly conserved gene among many of the species, encodes a highly conserved protein (92 kDa) that plays a central role in many metabolic processes, comprising cell cycle progression, cell proliferation, signaling transduction, and cell apoptosis. Current studies have conveyed that DEPDC1 has been involved in different types of human malignancies, like lung metastasis, bladder malignancy, nasopharyngeal malignancy, prostate cancer, and glioma [23]. Deoxyuridine monophosphate is transformed to deoxythymidine monophosphate, which is catalyzed by the thymidylate synthase, encoded TYMS. There is a chance of deoxynucleotide imbalance and increase in the levels of deoxyuridine monophosphate (dUMP) due to suppression of thymidylate synthase, resulting in damage of DNA [24]. Thymidylate synthase has been extensively used as a chemotherapeutic target recognized for its function in proliferation. In the study, experimental validation revealed TS as one of the highly ranked biomarkers identified. However, those chemotherapeutic drugs that target the enzyme might also appease other negative features related to carcinoma [25]. Fibronectin 1 (FN1) is a glycoprotein particle, which plays an important role in differentiation and migration, cell adhesion, cell growth, and wound repairing and embryonic development [26]. FN1 has been implicated to be a significant part in different threatening tumors such as lung cancer, colorectal malignant growth, and ovarian disease [27].

## 5. Conclusion

In conclusion, bioinformatics analysis of our study in breast cancer comes up with a worthy indication for biomarkers. BUB1, NCAPG, CHEK1, RACGAP1, SHCBP1, SDC1, CDC7, DEPDC1, TYMS, and FN1 were predicted as hub genes based on PPI analysis, and survival analysis was performed using the TCGA and KM plotter to validate the above results. Those major hub genes were found to be related with the risk of metastasis, and this finding would be taken out as future research. We hope that this research will provide some proof for future genetic personalized treatment in new perception for breast adenocarcinoma.

## Figures and Tables

**Figure 1:** Overall work plan for identification of strong prognostic biomarker genes in BAC.

**Figure 2:** Volcano plots: GPL4133 (a) and GPL13607 (b) expressions of the upregulated genes and downregulated genes. Upregulated genes are shown in red color, downregulated genes are shown in blue, and nonsignificant genes are shown in black with a log2 fold-change of 1.0 and an adjusted *p* value of 0.005.

**Figure 3:** The differentially expressed genes (DEGs) are displayed in heat maps: GPL4133 (a) and GPL13607 (b) with hierarchical grouping. High expression levels are addressed in red color, and lower expression levels are addressed in blue color.

**Figure 4:** The overlapping between two GEO data sets is shown by a Venn diagram. The Venn diagram indicates the overlaps in upregulated (a) and downregulated genes (b) in the given two data sets.

**Figure 5:** STRING network. This network contains 9 nodes and 20 edges, with a confidence score of 0.700, average node degree 1.54, average local clustering coefficient 0.303, and PPI enrichment *p* value 1.4e − 10. The pearl shape indicates the genes, the lines show the interaction of protein between the genes, and inside the circle is protein, and the color of the line represents the proof of interaction between the proteins.

**Figure 6:** Cytoscape software was used to retrieve the top hub genes. The node color gives an idea for the connection degree. The major ten hub genes show the color change from red to yellow. The red color represents the highest degree node, the light orange represents the intermediate one, and the yellow color reflects the lowest degree node among the top 10 hub genes.

**Figure 7:** Overall survival analysis of key genes in BAC patients, drawn by the KM plotter. The gene expression of the patients was classified into two groups based on the median high expression and low expression. The genes were (a–j) BUB1, NCAPG, CHEK1, RACGAP1, SHCBP1, SDC1, CDC7, DEPDC1, TYMS, and FN1 The survival curve shows the worse prognosis of BAC.

**Figure 8:** In GEPIA2, survey of the 10 key genes in the TCGA database. The box plot indicates the expression levels of the BAC genes, namely, (a–j) BUB1, NCAPG, CHEK1, RACGAP1, SHCBP1, SDC1, CDC7, DEPDC1, TYMS, and FN1.

**Figure 9:** (a–i) Correlation of the other BAC genes with BUB1 in GEPIA. NCAPG, CHEK1, RACGAP1, SHCBP1, CDC7, DEPDC1, and TYMS are positively correlated with BUB1.

**Table 1:** Gene Expression Omnibus provided evidence for the two expression profiles.

	Reference	Platform	Normal	Tumor
GSE70951	Quigley DA et al., 2017, update 2018	GPL4133 Agilent-014850 Whole Human Genome Microarray4x44k G4112F (Feature Number Version)	46	46

		GPL13607 Agilent-028004 SurePrint G3 Human GE 8x60k Microarray (Feature Number Version)	147	147

**Table 2:** Visualization of DEGs.

DEGs	Gene terms
Upregulated genes	ADAR, ARHGEF19, ATAD5, BFSP2, BUB1, C1QTNF6, C3orf14, C9orf116, CA12, CA14, CDC144NL, CD2, CD9, CDC7, CEACAM5, CHK1, COL5A2, COL7A1, CPA6, CRYM, CST2, DAPP1, DNASE1L2, DPP3, DQX1, DEPDC1, EGLN3, ETV7, FCHO1, FN1, FZD3, GLOD5, HGD, HOPX, ICOS, IGFL2, IGSF9, IL4I1, ITGB6, KCNF1, KIAA1522, KIAA1257, KIFC2, KIHL17, KREMEN2, LAG3, LHX2, LO145694, LOC283710, LY75, LYPD5, LYPLA1, MAGIX, MAPK13, MEI1, MMP7, MUC5B, NCAPG, NUS1AP, OASL, PAH, PARP9, PLA2G10, PRRT3, RAB17, RACGAP1, RALGPS2, RAMP1, RASAL, SDC1, SH2D2A, SHCBP1, SLC44A1, SLC44A3, SLC45A3, SNORA73A, STAG3, TCL1B, TEX19, TRAF4, TRIB3, TROAP, TYMS, UGT2B7, ZNF296.

Downregulated genes	ABI3BP, ACYP2, ADAMTS5, ADCY6, ADD1, ADRA1B, ALDH2, AMOYL2, ARHGAP20, MBDH2, MBMX, CALCOCO2, CCDC85A, CFH, CHST7, CLEC3B, CMTM2, CTDSP1, DCUN1D3, EFNB1EPS8, EYA4, FGFRL1, FNDC4, FUT4, FZD4, GPT2, H19, HIF3A, KATNAL1, KLHL10, LAMA2, LOC643802, LPL, ME1, MEOX2, MESP1, METTL7A, MFGE8, MMP27, MPDZ, MTMR10, MYL2, NEXN, NFIL3, NPR3, NQO2, PAX3, PHLDA3, PIK3R1, PLCD3, PODN, RADIL, RNF150, RNF180, RPS28, SCARA5, SCGN, SEMA3D, SGCA, SHC3, ST6GALNAC3, TLCD2, TMEM132C, TNMD, TUBB2B, UNC13B, ZBTB47, ZHX3, ZNF502.

**Table 3:** BC patient's overall survival and *p* value for top 10 regulatory genes in GSE70951.

Gene	HR (95% CI)	*p* value
BUB1	0.93 (0.84-1.02)	0.13
NCAPG	1.83 (1.65-2.03)	1*E* − 16
CHEK1	1.24 (1.07-1.44)	0.0048
RACGAP1	1.81 (1.64–2.01)	<1*E* − 16
SHCBP1	1.7 (1.53–1.88)	<1*E* − 16
SDC1	1.15 (1.04–1.27)	0.0073
CDC7	1.2 (1.08–1.33)	4*e* − 04
DEPDC1	1.59 (1.37–1.85)	1.4*e* − 09
TYMS	1.53 (1.38–1.7)	1.3*e* − 16
FN1	1.09 (0.98–1.21)	0.096

## Data Availability

The data used to support the findings of this study are available from the corresponding author upon request.

## Abbreviations

BAC: Breast adenocarcinoma
GO: Gene ontology
GEO: Gene Expression Omnibus
DEG: Differentially expressed gene
GEPIA: Gene Expression Profiling Interactive Analysis
KEGG: Kyoto Encyclopedia of Genes and Genomes
BP: Biological process
MF: Molecular function
CC: Cellular component
PPI: Protein-protein interaction
TCGA: The Cancer Genome Atlas
STRING: Search Tool for the Retrieval of Interacting Genes
BRCA: Breast Cancer gene
EMT: Epithelial-mesenchymal transition
NT: Normal tissue
DCIS: Ductal carcinoma in situ
BM: Basement membrane
MEC: Myoepithelial cell.
